# Improved Multiclassification of Schizophrenia Based on Xgboost and Information Fusion for Small Datasets

**DOI:** 10.1155/2022/1581958

**Published:** 2022-07-19

**Authors:** Wenjing Zhu, Shoufeng Shen, Zhijun Zhang

**Affiliations:** ^1^Department of Neurology, Affiliated Zhongda Hospital, Research Institution of Neuropsychiatry, School of Medicine, Southeast University, Nanjing 210009, China; ^2^Affiliated Mental Health Center & Hangzhou Seventh People's Hospital, Zhejiang University School of Medicine, Hangzhou 310000, China; ^3^College of Science, Zhejiang University of Technology, Hangzhou, Zhejiang 310023, China

## Abstract

To improve the performance in multiclass classification for small datasets, a new approach for schizophrenic classification is proposed in the present study. Firstly, the Xgboost classifier is introduced to discriminate the two subtypes of schizophrenia from health controls by analyzing the functional magnetic resonance imaging (fMRI) data, while the gray matter volume (GMV) and amplitude of low-frequency fluctuations (ALFF) are extracted as the features of classifiers. Then, the D-S combination rule of evidence is used to achieve fusion to determine the basic probability assignment based on the output of different classifiers. Finally, the algorithm is applied to classify 38 healthy controls, 16 deficit schizophrenic patients, and 31 nondeficit schizophrenic patients. 10-folds cross-validation method is used to assess classification performance. The results show the proposed algorithm with a sensitivity of 73.89%, which is higher than other classification algorithms, such as supported vector machine (SVM), logistic regression (LR), *K*-nearest neighbor (KNN) algorithm, random forest (RF), BP neural network (NN), classification and regression tree (CART), naive Bayes classifier (NB), extreme gradient boosting (Xgboost), and deep neural network (DNN). The accuracy of the fusion algorithm is higher than that of classifier based on the GMV or ALFF in the small datasets. The accuracy rate of the improved multiclassification method based on Xgboost and fusion algorithm is higher than that of other machine learning methods, which can further assist the diagnosis of clinical schizophrenia.

## 1. Introduction

Schizophrenia (SZ) is a serious mental illness that interferes with a person's ability to think clearly, manage emotions, make decisions, and relate to others [1]. The positive symptoms, such as hallucinations and delusions, can lead to suicidal or aggressive behavior, while negative symptoms and cognitive impairment lead to a decline in quality of life and social function; all these symptoms will cause tremendous human suffering and economic burden [2]. However, SZ is diagnosed on the basis of clinical evaluation of symptoms and functional, no objective diagnostic biomarker set. In addition, there are two main types of schizophrenia, which are called deficit schizophrenia (DS) and nondeficit schizophrenia (NDS) [3]. Deficit syndrome of schizophrenia, also called negative symptoms of schizophrenia, includes social withdrawal, loss of motivation, poverty of speech, and blunting of affect. Compared with NDS, DS has greater cognitive impairment, worse long-term prognosis, and lower recovery rates, which persist or are found even during psychotic remissions [4, 5]. Therefore, it is quite important to diagnose SZ accurately and discriminate the two subtypes of SZ from healthy control (HC), particularly the discrimination between the DS and NDS.

Classification is a machine learning algorithm where we get the labeled data as input and we need to predict the output into a class [6]. If there are two classes, then it is called binary classification [7]. If there are more than two classes, then it is called multiclass classification. Nowadays, classification algorithm is widely used in the medical diagnosis, especially in the field of mental disorders. Early published research applied support vector machines with radial basis function kernel method to classify 15 schizophrenic patients and 15 HCs based on the structural image of the hippocampal complex only with 63% classification accuracy [8]. With the rapid development of computational psychiatry, a growing body of classification approaches are applied to discriminate SZ in recent years, such as logistic regression (LR), support vector machine (SVM), neural network (NN), random forest (RF), extreme gradient boosting (XGBoost), and deep learning [9]. In the early studies, many researchers focused on the binary classification problem in SZ. Greenstein et al. proposed the logistic regress classifier to discriminate 99 SZ patients from 99 HCs with 73.7% accuracy [10]. Nieuwenhuis et al. proposed the SVM classifier to discriminate 128 SZ patients from 111 HCs and achieved an accuracy of 71.4% [11]. Thereby, in the past years, feature reduction approaches were discussed and applied to improve the performance of classification. Ershad and Hashemi proposed the dispelling reduction approaches [12], Juneja and his colleagues obtained the discriminative features by using SVD model and a novel multivariate feature selection algorithm [13]. However, the accuracy was not high enough based on the classical classification algorithms, which was usually less than 75%. Then, many new classifiers and feature selection approaches are proposed to improve the classification performance. Up to 2018, Wang et al. developed the SVM model to discriminate SZ from HCs and achieved an accuracy of 92.4% [14]. In 2020, Kim et al. proposed the feature reduction method when there are redundant or correlated features based on the FDR value and achieved an accuracy of 96.2% [15]. Patel et al. proposed a classification algorithm to discriminate SZ versus HCs by busing deep learning in fMRI, and the accuracy was 92% [16]. Nowadays, the binary classification is not a hard work in the field of mental disorders. However, there is not only one type of SZ, such as DS and NDS, which is more difficult to discriminate each other or from HCs. In order to solve this problem, multiple classification methods for schizophrenic subtypes are necessary.

Few previous literatures have reported multiclass classifications for different types of psychiatric patients, and most of these classifications used traditional machine learning methods such as SVM and LR. For examples, Zhu et al. proposed the SVM model to classify first-episode, drug-naive SZ, ultrahigh risk for psychosis and HC with the global balanced accuracy only 73.37% and the sensitivity only 68.42%, using the fivefold cross-validation method [17]. Soon afterwards, multiple classification methods have been explored, such as three SVM models to classify the SZ, bipolar disorder, and HC [18] and classify depression, bipolar disorder, and HC [19]; an SVM combined with recursive feature elimination was used to classify first-episode SZ, chronic SZ, and HC [20]. Unfortunately, almost all the accuracy rate of the multiclass classification is less than 70%. In addition, because of the poor coordination in psychiatric patients, the amount of imaging data is generally small, which leads to an accuracy far below 70%.

In recent years, deep learning is widely used in the pattern recognition. Zeng et al. proposed a deep discriminant autoencoder network to learn imaging site-shared functional connectivity features to discriminate SZ from normal subjects. In their work, the accuracy of 85% is achieved [21]. Oh et al. collected 873 structural MRI datasets and discriminate the SZ from normal subjects by using a deep convolutional neural network [22]. Srinivasagopalan et al. proposed a deep learning algorithm for diagnosing SZ [23]. These deep learning algorithms are based on the original image data, such as CNN and DNN. However, the original image data is usually quite difficult to obtain. Many deep learning algorithms on small dataset is usually overfitting. Therefore, the machine learning algorithms are more suitable to improve the performance of the classical classifiers.

To the best of our knowledge, there is no study to implement the multiclass classification of DS, NDS, and HC based on multimodal imaging data of schizophrenia. Therefore, in order to achieve multiclass classification of schizophrenia and obtain higher classification results in small data, a new classification algorithm is proposed in this paper. In this algorithm, GMV and ALFF are selected as the features to construct multiclassifier based on Xgboost, respectively. Then, the fused model is built to improve the accuracy for the small datasets. The D-S fusion model is used to combine the output from different classifiers to determine the probability assignment for different subtypes and HC. The rest of this paper is structured as follows. In Section 2, the Xgboost classifier is proposed to discriminate DS and NDS from HC and the fusion model is introduced to combine information of output. The results obtained by applying our model are shown in Section 3. In Section 4, the main contribution of this paper is summarized.

## 2. The Fused Classification Algorithm Based on Xgboost for Three-Class Classification

In this section, a fused classification algorithm is proposed to improve the accuracy for the small datasets. This algorithm is applied to discriminate the subtypes of SZ from HC. There are three labels (DS, NDS, and HC) that should be assigned to each collected subject. To solve this problem, an improved multiclassification algorithm is introduced. Firstly, Xgboost algorithm is applied to classify them, which is one of the most widely used machine learning algorithms in classification problems [24]. The classifiers are constructed based on the features of GMV or ALFF, which is extracted from fMRI data. Then, the fusion model is used to combine the output information of the different classifier to determine the probability assignment of each class. Finally, the test subject will be classified into the class with the maximum probability. The flow chart of the proposed algorithm is shown in Figure 1.

### 2.1. Classifier Based on the Xgboost Algorithm

The Xgboost algorithm is composed of many weak classification and regression trees (CARTs). Taking the *i*th dataset (*x*_*i*_,*y*_*i*_) as an example, *x*_*i*_ is the input variable with several attributes of fMRI data and *y*_*i*_ is the real value of the given subject. For example, *y*_*i*_ = (1, 0, 0) means the *i*th subject is HC, *y*_*i*_ = (0, 1, 0) means the *i*th subject is DS, and *y*_*i*_ = (0, 0, 1) means the *i*th subject is NDS.

Then, an Xgboost model can be mathematically expressed in the following form [25]:

(1) $$\begin{array}{c} {\hat{y}}_{i}=\overset{K}{\underset{k=1}{\sum }}f_{k}\left(x_{i}\right), \end{array}$$

where *K* is the number of the CARTs, *f*_*k*_ is the predicted value of each independent CART, and ${\hat{y}}_{i}$ is the predicted value with respect to input *x*_*i*_.

The additive training model of Xgboost can be expressed as

(2) $$\begin{array}{c} \left\{\begin{array}{c} {\hat{y}}_{i}^{\left(0\right)}=0,\\ {\hat{y}}_{i}^{\left(k\right)}=\overset{k}{\underset{t=1}{\sum }}f_{t}\left(x_{i}\right)={\hat{y}}_{k}^{\left(k-1\right)}+f_{k}\left(x_{i}\right), \end{array}\right. \end{array}$$

where ${\hat{y}}_{i}^{\left(k\right)}$ is the predicted value of the *k*th CART.

The objective function of Xgboost includes a loss function and regularization term, which is expressed as

(3) $$\begin{array}{c} \text{obj}=\overset{n}{\underset{i=1}{\sum }}l\left(y_{i},{\hat{y}}_{i}\right)+\overset{K}{\underset{k=1}{\sum }}\Omega \left(f_{k}\right), \end{array}$$

where $l\left(y_{i},{\hat{y}}_{i}\right)$ can be used to measure the error between predicted value and real value, *n* is the number of the subjects, and *Ω* is the regularization item to avoid overfitting.

The specific form of *Ω*(*f*_*k*_) of the *k*th CART is given as

(4) $$\begin{array}{c} \Omega \left(f_{k}\right)=\gamma T+\frac{1}{2}\lambda {\left\|w\right\|}^{2}, \end{array}$$

where *γ* and *λ* present the penalty coefficients, *T* is the number of leaf nodes, and *w* is the weight of the leaf nodes.

Then, the objective function of the *t*th step obj^(*t*)^ can be calculated by Equation (5) based on the previous step obj^(*t* − 1)^ based on the Equations (2) and (3).

(5) $$\begin{array}{c} \text{ob}{\text{j}}^{\left(t\right)}=\overset{n}{\underset{i=1}{\sum }}l\left(y_{i},{\hat{y}}_{i}^{\left(t-1\right)}+f_{t}\left(x_{i}\right)\right)+\overset{t-1}{\underset{k=1}{\sum }}\Omega \left(f_{k}\right)+\Omega \left(f_{t}\right). \end{array}$$

By applying the second-order Taylor expansion to above equation, the objective function can be transformed into

(6) $$\begin{array}{c} \text{ob}{\text{j}}^{\left(t\right)}=\overset{n}{\underset{i=1}{\sum }}l\left(y_{i},{\hat{y}}_{i}^{\left(t-1\right)}\right)+g_{i}f_{t}\left(x_{i}\right)+\frac{1}{2}h_{i}f_{t}^{2}\left(x_{i}\right)+\Omega \left(f_{t}\right)+\text{Const}. \end{array}$$

In the above expression, Const is a constant term at the step *t*; the parameters pair *g*_*i*_ and *h*_*i*_ can be calculated as

(7) $$\begin{array}{c} \left\{\begin{array}{c} g_{i}=\frac{\partial l\left(y_{i},{\hat{y}}_{i}^{\left(t-1\right)}\right)}{\partial {\hat{y}}_{i}^{\left(t-1\right)}},\\ h_{i}=\frac{\partial^{2}l\left(y_{i},{\hat{y}}_{i}^{\left(t-1\right)}\right)}{{\left(\partial {\overset{\wedge }{y}}_{i}^{\left(t-1\right)}\right)}^{2}}. \end{array}\right. \end{array}$$

Because$l\left(y_{i},{\hat{y}}_{i}^{\left(t-1\right)}\right)$is the constant item, the objective function can be rewritten as

(8) $$\begin{array}{c} \text{ob}{\text{j}}^{\left(t\right)}=\overset{n}{\underset{i=1}{\sum }}\left[g_{i}f_{t}\left(x_{i}\right)+\frac{1}{2}h_{i}f_{t}^{2}\left(x_{i}\right)\right]+\gamma T+\frac{1}{2}\lambda \overset{T}{\underset{j=1}{\sum }}w_{j}^{2}+{\text{const}}^{\prime }, \end{array}$$

where const′ is a new constant item at step *t*.

According to the definition of *f*_*k*_, *f*_*k*_ can be written in the following form as

(9) $$\begin{array}{c} f_{k}\left(x\right)=w_{q\left(x\right)}. \end{array}$$

Then, Equation (8) can be rewritten in the following form as

(10) $$\begin{array}{c} \text{ob}{\text{j}}^{\left(t\right)}=\overset{T}{\underset{j=1}{\sum }}\left[\left(\underset{i\in I_{j}}{\sum }g_{i}\right)w_{j}+\frac{1}{2}\left(\underset{i\in I_{j}}{\sum }h_{i}+\lambda \right)w_{j}^{2}\right]+\gamma T+{\text{const}}^{\prime }, \end{array}$$

denoted by∑_*i*∈*I*_*j*__*g*_*i*_ = *G*_*j*_and∑_*i*∈*I*_*j*__*h*_*i*_ = *H*_*j*_; then, the objective function is expressed as

(11) $$\begin{array}{c} \text{ob}{\text{j}}^{\left(t\right)}=\overset{T}{\underset{j=1}{\sum }}\left[G_{j}w_{j}+\frac{1}{2}\left(H_{j}+\lambda \right)w_{j}^{2}\right]+\gamma T+{\text{const}}^{\prime }. \end{array}$$

The leaf nodes of the *t*th CART are each independent; *G*_*j*_ and *H*_*j*_ are the determined items. Then, minimizing the function equation (11), the optimal parameter *w*_*j*_ can be calculated as

(12) $$\begin{array}{c} w_{j}^{*}=-\frac{G_{j}}{H_{j}+\lambda }. \end{array}$$

Therefore, the final objective function is shown in the following form as

(13) $$\begin{array}{c} {\text{obj}}^{*}=-\frac{1}{2}\overset{T}{\underset{j=1}{\sum }}\frac{G_{j}^{2}}{H_{j}+\lambda }+\gamma T+{\text{const}}^{\prime }. \end{array}$$

The splitting algorithm [26] based on the above function is used to find the best split in Xgboost by

(14) $$\begin{array}{c} \text{Gain}=\frac{1}{2}\left[\frac{G_{\text{L}}^{2}}{H_{\text{L}}+\lambda }+\frac{G_{\text{R}}^{2}}{H_{\text{R}}+\lambda }-\frac{{\left(G_{\text{L}}+G_{\text{R}}\right)}^{2}}{H_{\text{L}}+H_{\text{R}}+\lambda }\right]-\gamma . \end{array}$$

The gain function has four terms: the first two terms are the profits of left and right parts of a node, where *G*_L_ and *G*_R_ are the left and right parts of *G*_*j*_ and *H*_L_ and *H*_R_ are the left and right parts of *H*_*j*_; and the third item is the total profit of that node. The last item is the regularization item for preventing overfitting. The greedy algorithm determines whether a node obtains the maximum gain. Thus far, the optimal tree structure that maximizes the gain can be generated.

The above description leads to the split finding algorithm for Xgboost presented as Algorithm 1.

### 2.2. The Fusion Model Based on the D-S Evidence Theory

Analyses of the amplitude of low-frequency fluctuations (ALFF) and gray matter volume (GMV) are two important methods used in fMRI studies. Selecting GMV as the feature to construct the classifier based on the Xgboost algorithm, the predicted value of the *i*th subject can be obtained and denoted as ${\hat{y}}_{i}^{\left(1\right)}$, while the other predicted value ${\hat{y}}_{i}^{\left(2\right)}$can be calculated by selecting ALFF as the feature,${\hat{y}}_{i}^{\left(1\right)}\neq {\hat{y}}_{i}^{\left(2\right)}$usually. Taking the *i*th subject as an example, the output information of the classifiers is ${\hat{y}}_{i}^{\left(1\right)}=\left(0.7,0.3,0.9\right)$ and ${\hat{y}}_{i}^{\left(2\right)}=\left(0.7,0.5,0.6\right)$. According to the output of classifier based on the feature of GMV, this subject should be classified into NDS, while the classifier based on the feature of ALFF will classify this subject into HC.

To overcome the conflict of different classifiers, the D-S evidence model is used to fuse the information of ${\hat{y}}_{i}^{\left(1\right)}$ and ${\hat{y}}_{i}^{\left(2\right)}$ [27]. The softmax function [28] is used in many machine learning applications for multiclass classifications to assign probability for each subject. The softmax function is expressed in the following form as Equation (15), which is used to calculate the probability assignment of each class.

(15) $$\begin{array}{c} \left\{\begin{array}{c} {\hat{y}}_{ij}^{\left(1*\right)}=\frac{e^{{\overset{\wedge }{y}}_{ij}^{\left(1\right)}}}{\sum_{j=1}^{3}e^{{\overset{\wedge }{y}}_{ij}^{\left(1\right)}}},\\ {\hat{y}}_{ij}^{\left(2*\right)}=\frac{e^{{\overset{\wedge }{y}}_{ij}^{\left(2\right)}}}{\sum_{j=1}^{3}e^{{\overset{\wedge }{y}}_{ij}^{\left(2\right)}}}, \end{array}\right. \end{array}$$

where ${\hat{y}}_{ij}^{\left(1\right)}$ is the element in the set ${\hat{y}}_{i}^{\left(1\right)}$ and *j* = 1, 2, 3 represents HC, DS, and NDS, respectively. For example,${\hat{y}}_{i1}^{\left(1*\right)}$is the probability that the*i*th subject is HC according to the GMV feature, and${\hat{y}}_{i1}^{\left(2*\right)}$is the probability that the*i*th subject is HC according to the ALFF feature.

Though softmax function, the probability assignment of the *i*th subject can be obtained as

(16) $$\begin{array}{c} {\hat{y}}_{i}^{\left(1*\right)}=\left(0.3458,0.2318,0.4224\right),\\ {\hat{y}}_{i}^{\left(2*\right)}=\left(0.3672,0.3006,0.3322\right). \end{array}$$

Then, the combined strategy based on the D-S evidence is expressed as

(17) $$\begin{array}{c} \left\{\begin{array}{c} {\hat{y}}_{i}^{\left(1*\right)}⊕{\hat{y}}_{i}^{\left(2*\right)}\left(\text{HC}\right)=\frac{1}{K}\times {\hat{y}}_{i1}^{\left(1*\right)}\times {\hat{y}}_{i1}^{\left(2*\right)},\\ {\hat{y}}_{i}^{\left(1*\right)}⊕{\hat{y}}_{i}^{\left(2*\right)}\left(\text{DS}\right)=\frac{1}{K}\times {\hat{y}}_{i1}^{\left(1*\right)}\times {\hat{y}}_{i1}^{\left(2*\right)},\\ {\hat{y}}_{i}^{\left(1*\right)}⊕{\hat{y}}_{i}^{\left(2*\right)}\left(\text{NDS}\right)=\frac{1}{K}\times {\hat{y}}_{i1}^{\left(1*\right)}\times {\hat{y}}_{i1}^{\left(2*\right)}. \end{array}\right. \end{array}$$

The probability of subject into each group ${\hat{y}}_{i}^{\left(1*\right)}⊕{\hat{y}}_{i}^{\left(2*\right)}\in \left[0,1\right]$, where *K* reflects the conflict level of evidences and can be represented as

(18) $$\begin{array}{c} K={\hat{y}}_{i1}^{\left(1*\right)}\times {\hat{y}}_{i1}^{\left(2*\right)}+{\hat{y}}_{i1}^{\left(1*\right)}\times {\hat{y}}_{i1}^{\left(2*\right)}+{\hat{y}}_{i1}^{\left(1*\right)}\times {\hat{y}}_{i1}^{\left(2*\right)}. \end{array}$$

The result of the above example is ${\hat{y}}_{i}^{\left(1*\right)}⊕{\hat{y}}_{i}^{\left(2*\right)}=\left(0.3768,0.2068,0.4164\right)$ by Equation (17). According to the output of the fusion information, this subject will be classified into the class of NDS.

## 3. Experiments and Results

To evaluate performance of the proposed classification method, we scan 246 brain regions of 85 subjects by fMRI to extract the features of GMV and ALFF, including 16 DS, 31 NDS, and 38 HC. Obviously, it is a hard task to classify them in these small datasets. We apply the proposed algorithm to classify all the subjects.

The present study classifies all subjects into three classes by applying linear regression (LR), supported vector classifier (SVC), *K*-nearest Neighbor (KNN), neural network (NN), naive Bayes (NB), classification and regression tree (CART), random forest (RF), extreme gradient boosting (Xgboost), deep neural network (DNN), and the proposed fusion algorithm. The flow of 10-fold cross-validation is shown in Figure 2. The results of 10-fold cross-validation of different classifiers are shown as below.

The receiver operating characteristic (ROC) curve is considered to evaluate the performance of classifiers. For different classification thresholds, the true-positive rate (TPR) (Equation (19)) is plotted against the false-positive rate (FPR) (Equation (20)). The area under the ROC curve (AUC) indicates the classifier's ability to distinguish between classes. The value of the AUC is in the range [0,1]. AUC is 1 for a perfect classifier. In this work, the ROC curve is plotted for each class, as this is a multiclass problem. The microaverage and macroaverage are also computed by summing the individual values for true positive (TP), true negative (TN), false positive (FP), and false negative (FN). Then, the accuracy (Equation (21)), recall (Equation (22)), precision (Equation (23)), and F1-score (Equation (24)) are selected as the important metrics to evaluate the performance of different classifiers [29].

(19) $$\begin{array}{c} \text{TPR}=\frac{\text{TP}}{\text{TP}+\text{FN}}, \end{array}$$

(20) $$\begin{array}{c} \text{FPR}=\frac{\text{FP}}{\text{FP}+\text{TN}}, \end{array}$$

(21) $$\begin{array}{c} \text{Accuracy}=\frac{\text{TP}+\text{TN}}{\text{TP}+\text{TN}+\text{FP}+\text{FN}}, \end{array}$$

(22) $$\begin{array}{c} \text{Precision}=\frac{\text{TP}}{\text{TP}+\text{FP}}, \end{array}$$

(23) $$\begin{array}{c} \text{Recall}=\frac{\text{TP}}{\text{TP}+\text{FN}}, \end{array}$$

(24) $$\begin{array}{c} \text{F}1‐\text{score}=\frac{2\times \text{precision}\times \text{recall}}{\text{precision}+\text{recall}}. \end{array}$$

The ROC of the above classifiers are shown in Figures 3–8. In these figures, DS is the class 0, HC is the class 1, and NDS is the class 2. The key classification metrics are extracted from the results listed in Table 1.

Due to the limited number of the DS, the AUC of class 0 is lower than other classes in the above figures. Therefore, it is hard to discriminate DS from NDS and HC. Taking Figure 5 as an example, the macroaverage AUC score is 0.81 and the microaverage AUC score is 0.85 based on the feature of GMV by using the SVM classifier, which are better than the performance based on the feature of ALFF. The AUC score of HC is 0.85 based on the feature of GMV, which is better than the AUC scores of DS and NDS. The Xgboost classifier showed better performance than the SVM and logistic classifier. The microaverage AUC score is 0.90 and 0.80, respectively, on the feature of GMV and ALFF. The macroaverage AUC score is 0.90 and 0.84, respectively, on the feature of GMV and ALFF. The ROC of the fusion algorithm is shown in Figure 9. In this figure, we find the AUC score of the class 0 is 1, which means it is a perfect classifier. This classifier combines the advantages of the classifier based on feature of GMV and ALFF. Therefore, the performance of this fusion classifier is much better than others.

From Table 1, 10-fold cross-validation showed our algorithm with an accuracy of 73.89%, which is higher than other classifiers. Many metrics of the proposed classifier are better than other classifiers. In many present studies, the accuracy of the present classifier is usually less than 70% when the datasets are small. In this paper, the proposed fusion classifier will improve the performance effectively for the small datasets by combining the advantages of each feature. The accuracy of different classifiers is shown in Figure 10.

## 4. Conclusion

In this paper, a new multiple classifier method was proposed for the small datasets and applied to discriminate the two subtypes of schizophrenia and health controls based on the fMRI data. Due to the limitation data and indexes, this study constructed the Xgboost algorithm based on the different features. To improve the accuracy, the fusion model was used to combine the information from different classifiers. Finally, the subject would be classified into the class with the maximum probability. This method was applied to classify 38 healthy controls, 16 deficit schizophrenic patients, and 31 nondeficit schizophrenic patients. 10-fold cross-validation showed our algorithm with a sensitivity of 73.89%, which was much higher than other classification algorithms when the datasets were small. In addition, the proposed algorithm can be used to discriminate different classes for the large datasets. The performance of the proposed algorithm would be effective than other algorithms when the datasets are small. It will bring the better performance in diagnosing subtypes of schizophrenia. Although the findings in our study are rigorous, there are some limitations: (1) relatively small sample size; (2) interference caused by antipsychotic drugs during experiment; and (3) limitations of the algorithm itself. In the future work, more subjects will be collected in the project, including different subtypes and HC. The original image data should be obtained in the processing of experiments, and more deep learning approaches will be proposed to solve this multiclass classification problem.

## Figures and Tables

**Figure 1:** Flow chat of improved multiclassification algorithm.

**Figure 2:** Flow chat of 10-fold cross-validation.

**Figure 3:** Results of logistic classifier (GMV).

**Figure 4:** Results of logistic classifier (ALFF).

**Figure 5:** Results of SVM with kernel of RBF (GMV).

**Figure 6:** Results of SVM with kernel of RBF (ALFF).

**Figure 7:** Results of Xgboost (GMV).

**Figure 8:** Results of Xgboost (ALFF).

**Figure 9:** Results of Xgboost (fusion).

**Figure 10:** Accuracy of different classifiers.

**Algorithm 1:** Greedy algorithm for split finding.

**Table 1:** Classification metrics of different methods.

Methods	Accuracy	Precision	Recall	F1-scores	AUC
LR (GMV)	64.8611%	65.0509%	64.8611%	0.6237	0.8160
LR (ALFF)	65.9722%	65.5394%	65.9722%	0.6388	0.7743
SVC (GMV)	61.5278%	51.5602%	61.5277%	0.5508	0.7403
SVC (ALFF)	67.0833%	59.4147%	67.0833%	0.6114	0.6114
KNN (GMV)	63.4722%	61.4259%	63.4722%	0.5899	0.7174
KNN (ALFF)	58.6111%	67.3175%	58.6111%	0.5601	0.6731
NN (GMV)	55.4167%	56.4749%	47.2222%	0.5425	0.8066
NN (ALFF)	64.4444%	67.0764%	60.8333%	0.6266	0.7618
NB (GMV)	53.8889%	55.8657%	53.8889%	0.5216	0.7389
NB (ALFF)	68.8889%	74.0139%	68.8889%	0.6781	0.8308
CART (GMV)	45.8333%	47.7870%	51.9444%	0.4721	0.6375
CART (ALFF)	60%	57.6075%	56.6667%	0.5667	0.6542
RF (GMV)	62.6389%	60.0883%	62.6389%	0.5874	0.7722
RF (ALFF)	65.6944%	57.1042%	65.6944%	0.5943	0.7969
Xgboost (GMV)	62.6389%	60.4445%	62.6389%	0.5888	0.7958
Xgboost (ALFF)	68.0556%	62.9610%	68.0556%	0.6364	0.8351
DNN	62.7083%	40.3380%	62.7083%	0.5152	0.6723
Our classifier (fusion)	73.8889%	65.4242%	73.8889%	0.6746	0.8524

## Data Availability

No data were used to support this study.
